The article "Isovitexin reduces carcinogenicity and stemness in hepatic carcinoma stem-like cells by modulating MnSOD and FoxM1" was retracted in 2022. Reasons: duplicated images; original data or images not available; unreliable data.

# Isovitexin reduces carcinogenicity and stemness in hepatic carcinoma stem-like cells by modulating MnSOD and FoxM1

**DOI:** 10.1186/s13046-019-1244-6

**Published:** 2019-06-17

**Authors:** Xiaocheng Cao, Lihua Liu, Qing Yuan, Xiang Li, Yinghong Cui, Kaiqun Ren, Chang Zou, A. Chen, Chang Xu, Yebei Qiu, Meifang Quan, Jiansong Zhang, Jianguo Cao, Xiangding Chen

**Affiliations:** 1 Department of Pharmaceutical Science, Medical College, Hunan Normal University, Changsha, 410013 Hunan China; 2 Key Laboratory of Study and Discover of Small Targeted Molecules of Hunan Province, Changsha, 410013 Hunan China; 3 Laboratory of Molecular and Statistical Genetics, College of Life Sciences, Hunan Normal University, Changsha, 410081 Hunan China; 4 Pharmacy Department, the Second Clinical Medical School of Jinan University, Shenzhen People’s Hospital, Shenzhen, 518020 China; 5 Shenzhen Public Service Platform on Tumor Precision Medicine and Molecular Diagnosis, Shenzhen People’s Hospital, Shenzhen, 518020 China; 6 Department of Preclinical Medicine, Medical College, Hunan Normal University, Changsha, 410013 Hunan China; 7 Clinical Medical Research Center, the Second Clinical Medical School of Jinan University, Shenzhen People’s Hospital, Shenzhen, 518020 China

**Keywords:** Hepatic carcinoma, **C**ancer stem cells, Isovitexin, MnSOD, FoxM1

## Abstract

**Background:**

Manganese superoxide dismutase (MnSOD) upregulating FoxM1 have previously been demonstrated promoting lung cancer stemness. Isovitexin exhibits antitumor activities in various cancers. This study aimed to assess whether isovitexin inhibits hepatic carcinoma stem-like cells (HCSLCs) features via regulating MnSOD and FoxM1 expression.

**Methods:**

Second-generation spheres from the hepatic carcinoma cell lines, respectively, were used as HCSLCs. Protein amounts of MnSOD, FoxM1 and stemness-associated markers (CD133, CD44, ALDH1, Bmi1, Nanog and Oct4) were determined by immunoblotting. In vitro carcinogenicity was evaluated by sphere- and colony-formation assays. The effects of isovitexin on HCSLC carcinogenicity and stemness were examined in vitro and in xenograft models. An adenoviral delivery system was employed to manipulate MnSOD and/or FoxM1. Luciferase reporter assay was performed to verify isovitexin downregulated FoxM1 by inhibiting MnSOD-mediated effects of E2F1 and/or Sp1 on activation of FoxM1 promoter.

**Results:**

FoxM1 upregulation by MnSOD contributed to carcinogenicity and stemness, with increased sphere- and colony-formation capabilities, upregulated stemness-associated markers and CD133^+^ subpopulation as well as elevated oncogenicity in vivo in HCSLCs compared with hepatic carcinoma cells. Isovitexin substantially decreased sphere and colony formation rates, and stemness-associated markers in cultured HCSLCs by suppressing MnSOD and FoxM1 expression. Importantly, isovitexin significantly inhibited tumor growth of in nude mice bearing HCSLCs and reduced CD133 protein expression of xenograft in nude mice. MnSOD or FoxM1 knockdown enhanced the effects of isovitexin suppression on carcinogenicity and stemness in HCSLC. MnSOD or FoxM1 overexpression attenuated the effects of isovitexin. Additionally, isovitexin and MnSOD knockdown could inhibit FoxM1 reporter activity via a decreased binding of E2F1 and/or Sp1 onto FoxM1 promoter. FoxM1 overexpression reversed the effects of isovitexin combined with MnSOD knockdown, without affecting MnSOD expression. Moreover, MnSOD knockdown plus thiostrepton, a FoxM1 specific inhibitor, cooperated with isovitexin to repress xenograft tumor growth and downregulate MnSOD and FoxM1 in nude mice bearing HCSLCs from MHCC97H cells.

**Conclusions:**

Isovitexin inhibits carcinogenicity and stemness in HCSLCs by downregulating FoxM1via inhibition of MnSOD.

**Electronic supplementary material:**

The online version of this article (10.1186/s13046-019-1244-6) contains supplementary material, which is available to authorized users.

## Background

Human hepatic carcinoma is tightly associated with high incidence and mortality owing to recurrence and metastasis after current routine treatments [1]. Hepatic carcinoma stem-like cells (HCSLCs) are mainly contributor to poor prognosis in hepatic carcinoma patients because of a high potential for tumor initiation, progression, recurrence and metastasis [2, 3]. Therefore, targeting putative HCSLCs may be an effective therapeutic strategy for human hepatic carcinoma treatment [4].

Currently, Forkhead box M1 (FoxM1) is considered a carcinogenic transcription factor, which is substantially elevated in the majority of human cancers, including hepatic carcinoma [5, 6]. Knockdown of FoxM1 leads to cell-cycle arrest and mitotic catastrophe [7, 8]. FoxM1 is abnormally upregulated in human hepatic carcinoma tissues, with its overexpression involved in poor prognosis of hepatic carcinoma patients [9–12]. Deletion of FoxM1 in mouse hepatocytes results in inhibited cell proliferation and reduced hepatic carcinoma development in response to diethyl-nitrosamine [13]. We and others reported that overexpression of manganese superoxide dismutase (MnSOD) could upregulate FoxM1 to promote invasion and migration in NSCLC and lung cancer stem-like cells [14, 15]. However, whether FoxM1 upregulation by MnSOD maintains carcinogenicity and stemness in HCSLCs, thereby stimulating tumor development and progression, as well as the significance of its modulation on targeting HCSLCs for hepatic carcinoma treatment remain unknown.

MnSOD under physiological conditions is a substantial redox-enzyme localized to the mitochondrial matrix, and converts the mitochondrial product superoxide anion radical into hydrogen peroxide (H_2_O_2_) to regulate cellular signal transduction [16]. The antioxidant function of MnSOD is considered to be tumor suppressive, which may reduce carcinogenicity in several cancers, including pancreatic cancer [17], colorectal cancer [18] and multiple myeloma [19]. Conversely, abnormal expression of MnSOD in certain cancers, such as gastric cancer [20], cervical cancer [21] and lung cancer [22], may promote carcinogenicity and disease progression. Our recent study demonstrated that MnSOD overexpression confers carcinogenicity and stemness to NCI-H460 cell line [15]. However, its effects on carcinogenicity and stemness in HCSLCs remain unclear.

Isovitexin (apigenin-6-C-glucoside) possesses high resistance to acid hydrolysis due to C-6 forming a C–C bond, thereby exerting a wide range of biological activities [23, 24]. We and others revealed isovitexin as an active constituent of the fruits of *Cucurbitaceae*, *Vigna radiata* and *Vitex trifolia L*. [25, 26], which exhibits antitumor activities by inducing cell apoptosis in HepG2, HeLa and HCT116 cells [27–29]. Our previous work demonstrated that Fructus Viticis total flavonoids (FVTF), an active fraction containing isovitexin selectively suppress tumor sphere forming capacity as well as migration and invasion in lung cancer stem-like cells derived from NCI-H446 cells [26]. In preliminary studies, we found that isovitexin significantly inhibits sphere- and colony-forming capabilities, accompanied by parallel downregulation of MnSOD and FoxM1 at the protein level in HCSLCs. Therefore, this study aimed to assess whether isovitexin inhibits carcinogenicity and stemness in HCSLC and explore the potential mechanisms.

## Methods

### Sphere culture

For sphere formation, human hepatocellular carcinoma MHCC97H and SMMC-7721, and hepatoblastoma HepG2 cells obtained from the Cell Bank of Chinese Academy of Sciences (Shanghai, China; 10,000 cells/well) were devoid of serum and cultured in DMEM/F12 (Invitrogen, Carlsbad, CA, USA) with 2% B27 (Invitrogen), 20 ng/ml EGF (Invitrogen), 20 ng/ml bFGF (Invitrogen), 4 μg/ml insulin (Sigma-Aldrich), 100 IU/ml penicillin G and 100 μg/ml streptomycin (cancer stem cell conditioned medium, CSC-CM), and plated into ultra-low attachment 6-well plates (Corning Inc., Corning, NY, USA). This was followed by incubation for 6 days to obtain the first-generation spheres, which were further subjected to sphere culture to yield second-generation spheres used as HCSLCs. Next, HCSLCs were incubated without or with various concentrations (5, 10 and 20 μM) of isovitexin (Sigma-Aldrich St., Louis, MO, USA) for 72 h in fresh CSC-CM.

To determine the sphere-forming rate, MHCC97H, SMMC-7721 and HepG2 cells or respective HCSLCs incubated with or without isovitexin (Sigma-Aldrich) were disintegrated into single cells resuspended in CSC-CM and seeded into ultra-low attachment 24-well plates (Corning Inc.) at 1 × 10^3^ cells/well. After 6 days of incubation, spheres were counted, and the sphere-forming rate (%) was determined by dividing the total number of spheres obtained by that of live cells seeded, multiplied by 100.

### Colony formation assay

The bottom layer was prepared by mixing 1.6% agarose (Invitrogen) with DMEM (1:1; *v*/*v*) and adding the mixture into 24-well cell culture plates (500 μL) for 10 min until solidification. Then, the top layer containing MHCC97H, SMMC-7721 or HepG2 cells or respective HCSLCs (500 cells) incubated with or without isovitexin and 0.4% agarose (Invitrogen) in 500 μL of 20% FBS DMEM were placed over the bottom layer. Colonies were counted under an inverted microscope (Olympus CK40; Olympus Corp., Tokyo, Japan) after incubation at 37 °C for 21 days. The colony formation rate (%) was determined by dividing the number of colonies by that of cells seeded, multiplied by 100%.

### Immunoblot

Immunoblot was performed as previously described [26]. MHCC97H, SMMC-7721 and HepG2 cells or respective HCSLCs (5 × 10^5^ cells) were lysed on ice with RIPA Lysis buffer (Beyotime Institute of Biotechnology, Shanghai, China) containing 1% phenylmethylsulfonyl-fluoride (PMSF; Sigma-Aldrich St.). Equal amounts (60 μg) of protein were separated by sodium dodecyl sulfate polyacrylamide gel electrophoresis (SDS-PAGE) and transferred onto polyvinylidene fluoride (PVDF) membranes (Millipore, Billerica, MA, USA). After blocking with 5% non-fat milk, the membranes were incubated with anti-β-actin (Catalog No. A5441; Sigma-Aldrich), anti-MnSOD (Catalog No. ab13533; Abcam, Cambridge, MA, USA), anti-FoxM1 (Catalog No. sc-502; Santa Cruz Biotechnology, Inc., Beverly, MA, USA) and anti-CD133, anti-CD44, anti-ALDH1, anti-Bmi1, anti-Nanog and anti-Oct4 (Catalog No. 5860S, 3570S, 12035S, 5855S, 3580S and 2788S; Cell Signaling Technology, Danvers, MA, USA) primary antibodies overnight at 4 °C, followed by incubation with appropriate HRP-conjugated secondary antibodies (Beyotime Institute of Biotechnology, Shanghai, China) for 1 h at room temperature. Immunoreactive bands were visualized using an enhanced chemiluminescence detection system (Ranon GIS-2008, Tanon Science & Technology Co., Ltd., Shanghai, China). Immunoblots were scanned and semi-quantitated with the Image Pro-Plus 6.0 software (Media Cybernetics, Rockville, MD, USA).

### Flow cytometry (FCM) analysis of CD133 expression

MHCC97H cells (1 × 10^6^) or HCSLCs (1 × 10^6^) treated with or without isovitexin (5, 10 and 20 μM) were incubated with William’s E medium supplemented with 20% FBS for 30 min in ambient conditions for blocking. After two PBS washes, the cells were resuspended in 990 μl PBS, and administered 10 μl of PE-linked anti-CD133 or isotype control IgG2b (Biolegend) for 30 min at 4 °C away from light. Upon fixation with 0.1% formaldehyde, analysis was performed on a FACS Calibur™ system (BD, USA).

### Adenovirus and infection

Transduction of MnSOD- and FOXM1-targeted shRNAs or overexpression plasmids was carried out as previously described [15]. Briefly, MHCC97H cells and/or HCSLCs were transferred into 100 mm petri dishes (Corning Inc.) at 40-50% confluence and incubated overnight. Cells were then infected with pHBad-MCMV-GFP, pHBad-U6-GFP, pHBad-MCMV-GFP-MnSOD, pHBad-MCMV-GFP-FoxM1, pHBad-U6-GFP-sh MnSOD and pHBad-U6-GFP-sh FOXM1 plasmid packaging adenoviral particles (Hanbio Biotechnology Co. Ltd., 2.0 mL, 1 × 10^11^ PFU/ mL; Shanghai, China) with the enhanced infection solution (ENi.s; GeneChem, Catalog No.REVG0002, Shanghai, China) in Opti-MEM (Invitrogen) for 2 h, respectively, at a MOI (multiplicity of Infection) of 100. After infection, the medium was replaced with DMEM containing 10% FBS. Infection efficiency was assessed by counting GFP-positive and live cells under an inverted fluorescent microscope (Olympus CK40; Olympus Corp.).

### Luciferase reporter assay of FOXM1 promoter fragment

Human FOXM1 promoter fragment (from − 330 to + 26) that contain E2F1 and Sp1 putative binding sites were amplified from human genomic DNA (Roche Company, Basel, Switzerland) using TaKaRa LA Taq, and inserted into the pGL3-Basic luciferase reporter vector (Promega, Madison, WI, USA). HCSLCs derived from MHCC97H cell line with or without transduction of MnSOD shRNA or treatment of isovitexin were co-transfected with 200 ng FOXM1 luciferase promoter or pGL3-Basic as control and pRL-TK (Promega) encoding Renilla luciferase was used as an internal control (10 ng/well) to assess transfection efficiency. Then, cells were lysed and assessed with the dual luciferase reporter assay system (Promega) as directed by the manufacturer. *Renilla* luciferase activity was employed for normalization, and triplicate assays were repeated three times.

### In vivo xenograft studies

Male BALB/c-nu mice (12-14 g) aged 30 days obtained from Nanjing Institute of Biomedical Research at Nanjing University were assessed. All mouse experiments were approved by the Ethics Committee of Hunan Normal University, and experimental protocols were performed in accordance with the Board of Laboratory Animal Feeding and Use Management Committee.

For in vivo tumorigenicity assay, mice (*n* = 4) were subcutaneously injected HCSLCs (1 × 10^3^) into the left flank, with the corresponding MHCC97H cells (1 × 10^5^) in the right flank, respectively. After 2 month, the mice were euthanized and xenografts were weighed after extraction since the largest diameters exceeded 1.5 cm of HCSLC xenografts. Xenograft specimens were fixed in 10% neutral formalin. Tissue sections were submitted to H&E staining, with histopathological morphology evaluated by optical microscopy.

To estimate the effects of isovitexin in the xenograft mouse model, HCSLCs from MHCC97H cells (2 × 10^6^/ml) suspended in CSC-CM were mixed with matrigel (1:1; BD Biosciences, San Jose, CA, USA), and 100 μL mixture of the was injected subcutaneously into each BALB/c-nu mouse. When the xenograft volume reached about 200 mm^3^, the mice were administered 200 μl of vehicle [30% captisol (Selleck Chemicals, Houston, TX, USA) in water: 5% glucose (1:1 V/V)] in the control group, or isovitexin (10, 20 and 40 mg/kg body weight, respectively) by gavage every 2 days for a total of 7 times. There were 4 mice in each treatment group.

To determine whether isovitexin-associated inhibition of xenograft tumor growth is involved in FoxM1 upregulation by MnSOD, HCSLCs from MHCC97H cells (2 × 10^6^) in CSC-CM were mixed with matrigel (1:1; BD Biosciences), and 100 μL of the mixture was injected subcutaneously into each BALB/c-nu mouse. When the xenograft volume reached 50 mm^3^, the mice were administered 200 μl of vehicle [30% captisol (Selleck Chemicals) in water: 5% glucose (1:1; V: V)] in the control group; oral isovitexin dissolved in 200 μl of vehicle (20 mg/kg), every other day for a total of 7 times, was administered to the isovitexin group; intratumorally injection with 20 μL per mouse of adenovirus expressing MnSOD shRNA (Hanbio Biotechnology Co. Ltd.), once a week for 2 week, was performed for the MnSOD knockdown group; oral treatment with the FOXM1 specific inhibitor thiostrepton (5 mg/kg in 200 μl of vehicle) once on alternate days, was performed for a total of 7 times as in the thiostrepton group; injection of the adenovirus expressing MnSOD shRNA plus isovitexin combined with thiostrepton was carried out in the combination group. There were 6 mice in each group. Then, the longest (L) and shortest (W) diameters of the subcutaneous xenografts were measured with a Vernier caliper for volume assessment, according to the formula: V (transplanted tumor volume, mm3) = L × (W)^2^ × 0.5. At the end of the experiment, the animals were euthanized, and xenografts were weighed after extraction. Xenograft specimens were fixed with 10% neutral formalin. Tissue sections were submitted to H&E staining, and histopathological morphology was evaluated by optical microscopy.

### Immunohistochemistry

Tumor tissues were fixed with neutral phosphate buffer containing 4% formaldehyde (ICM Pharma, Pte Ltd., Kaliang place, Singapore) at room temperature for 24 h, processed by graded ethanol, and embedded in paraffin. Five μm sections were deparaffinized in xylene, rehydrated with graded concentrations of ethanol, and stained with hematoxylin and eosin solution (Sigma Diagnostics, St. Louis, Missouri, USA). For immunostaining, the standard Elivision plus method was performed with the Elivision plus kit (Maixin-Bio, Fuzhou, China). Primary antibodies [anti-MnSOD (Abcam) or anti-FoxM1 (Santa Cruz Biotechnology, Inc.) or anti-CD133 (Cell Signaling Technology) antibody] were applied at 1:200 dilution. For negative controls, phosphate-buffered saline (PBS) was used instead of the primary antibody to detect nonspecific reactions or false positives. Images were acquired under an Olympus BX60 microscope (Olympus, Japan).

### Statistical analysis

Data were analyzed with SPSS 20.0 for Windows (SPSS Inc., Chicago, USA). All experiments were repeated three times, and data are mean ± standard deviation (SD). Two-tailed Student’s *t*-test was used for group pair comparisons. Multiple groups were compared by one-way analysis of variance (ANOVA). First, homogeneity of variance was determined, and all pairwise comparisons between groups were analyzed by the least significant difference (LSD) method. The Tukey’s test was performed in case of incomplete variance for both the control and experimental groups. Statistical significance was determined as *p* < 0.05.

## Results

### Isovitexin represses carcinogenicity and stemness in HCSLCs from MHCC97H cells

We initially assessed whether the second generation spheres of MHCC97H cells could be used as HCSLCs. Immunoblot data indicated increased expression amounts of MnSOD and FoxM1 in HCSLCs compared with MHCC97H cells (Fig. 1a, Additional file 1: Figure S1a). Meanwhile, sphere and colony formation capabilities were potentiated in HCSLCs (Fig. 1b and c, Additional file 1: Figure S1b and c). Furthermore, the expression amounts of stemness-related markers (CD133, CD44, ALDH1, Bmi1, Nanog and Oct4) were increased in HCSLCs compared with MHCC97H cells (Fig. 1d, Additional file 1: Figure S1d). Importantly, the percentage of CD133^+^ cells was higher in the second generation spheres than MHCC97H cells and the third or fourth generation spheres (Fig. 1e, Additional file 1: Figure S1e).

**Fig. 1:** Isovitexin inhibits carcinogenicity and stemness in HCSLCs. **a** Immunoblotting performed with anti-MnSOD and anti-FoxM1 antibodies, with β-actin antibodies used as a loading control; **b** and **c** Formed spheres and colonies (Scale bar, 200 μm); **d** Immunoblotting for CD133, CD44 and ALDH1, Bmi1, Nanog and Oct4; **e** CD133^+^ cell population in MHCC97H cells and HCSLCs. **f** Decreased the amounts of MnSOD and FoxM1 in HCSLCs from MHCC97H cells following treatment with isovitexin (ISOV: 5.0, 10.0 and 20.0 μM). Isovitexin induced reduction of spheroid formation (**g**, Scale bar, 200 μm), colony formation (**h**, Scale bar, 200 μm), and protein amounts of CD133, CD44, ALDH1 and Bmi1, Nanog and Oct4 (**i**), CD133^+^ cell population (**j**) in HCSLCs

To compare carcinogenicity between HCSLCs (second generation spheres) and MHCC97H cells, HCSLCs (1 × 10^3^) and MHCC97H cells (1 × 10^5^) were inoculated into the left and right flanks of nude mice, respectively. The xenograft tumors of HCSLCs were larger and heavier than those of MHCC97H cells although HCSLC number was 1/100 that of MHCC97H cells (Additional file 1: Figure S1f). In addition, H&E staining revealed that the histological features of xenograft tumors in the HCSLC group were similar to those of MHCC97H Cells, but its cancer stem marker CD133 protein expression upregulation (Additional file 1: Figure S1f). These results demonstrate that second generation spheres from MHCC97H cells possessed HCSLC properties, which might be associated with MnSOD and FoxM1 overexpression.

To determine whether isovitexin inhibits carcinogenicity and stemness in HCSLCs from MHCC97H cells, we next assessed the sphere and colony formation abilities as well as the protein amounts of stemness-related markers after isovitexin treatment. The results showed that treatment of HCSLCs with isovitexin markedly decreased the protein levels of MnSOD and FoxM1 (Fig. 1f, Additional file 1: Figure S1g). In addition, isovitexin obviously reduced the sphere and colony formation capabilities (Fig. 1g and h, Additional file 1: Figure S1h and i). Furthermore, the protein amounts of CD133, CD44, ALDH1, Bmi1, Nanog and Oct4 were decreased by isovitexin treatment, in dose-dependent manner (Fig. 1i, Additional file 1: Figure S1j). Importanly, isovitexin significantly decreased the CD133^+^ cell percentage of HCSLCs, in a dose-dependent manner (Fig. 1j, Additional file 1: Figure S1k). These data suggested that isovitexin exerted suppression on carcinogenicity and stemness in HCSLCs from MHCCH cells, which might be associated with MnSOD and FoxM1 downregulation.

To determine whether isovitexin inhibits xenograft tumor growth of HCSLCs from MHCC97H cells in nude mice, mice bearing HCSLC tumors were orally treated every 2 days with 200 μl of vehicle, and 10, 20 and 40 mg/kg isovitexin, respectively, for 3 weeks. The results showed that oral delivery of isovitexin led to significantly reduced tumor growth and cancer stem marker CD133 protein expression, in a dose-dependent manner (Additional file 1: Figure S1l). These results confirmed isovitexin could effectually inhibit tumor growth and HCSLC properties of HCSLCs in vivo.

### Isovitexin-associated inhibition of carcinogenicity and stemness is affected by MnSOD expression alteration in HCSLCs from MHCC97H cells

To determine the role of MnSOD in the maintenance of carcinogenicity and stemness, we first knocked down MnSOD in HCSLCs by transduction with MnSOD shRNA (Additional file 2: Figure S2a). The results showed notably decreased protein amounts of MnSOD and FoxM1 in HCSLCs expressing MnSOD shRNA compared with non-transduced cells or the vector control group (Fig. 2a, Additional file 2: Figure S2b). In addition, sphere and colony formation capabilities of HCSLCs expressing MnSOD shRNA were significantly reduced (Fig. 2b and c, Additional file 2: Figure S2c and d). Furthermore, the expression amounts of CD133, CD44 and ALDH1 as well as Bmi1, Nanog and Oct4 in MnSOD knockdown HCSLCs were also reduced (Fig. 2d, Additional file 2: Figure S2e). Chen et al. reported that MnSOD overexpression in lung cancer cells promoted binding of E2F1 and Sp1 to their putative FoxM1 promoter-binding sites and activated FoxM1 reporter activity. We also found that the relative luciferase activity of FOXM1 promoter fragment (from − 330 to + 26) that contain E2F1 and Sp1 putative binding sites was reduced in HCSLCs expressing MnSOD shRNA compared with non-transduced cells or the vector control group (Fig. 2e).

**Fig. 2:** Effects of MnSOD shRNA or cDNA transduction on carcinogenicity and stemness in HCSLCs or MHCC97H cells. HCSLCs were transduced with Ad-GFP or Ad-shMnSOD. **a** Immunoblotting performed with anti-MnSOD and anti-FoxM1 antibodies, with β-actin antibodies used as a loading control; **b** and **c** Formed spheres and colonies (Scale bar, 200 μm); **d** Immunoblotting for CD133, CD44 and ALDH1, Bmi1, Nanog and Oct4; **e** The relative luciferase activity of FOXM1 promoter fragment in HCSLCs untreated (Mock), or transduced with Ad-GFP and Ad-sh MnSOD, respectively. MHCC97H cells were transduced with Ad-GFP or Ad-MnSOD. **f** Immunoblotting performed with anti-MnSOD and anti-FoxM1 antibodies; β-actin antibodies were used as a loading control; **g** and **h** Formed spheres and colonies (Scale bar, 200 μm); **i** Immunoblotting for CD133, CD44, ALDH1, Bmi1, Nanog and Oct4; **j** The relative luciferase activity of FOXM1 promoter fragment in MHCC97H cells untreated (Mock), and transduced with Ad-GFP and Ad-MnSOD, respectively

We next forced MnSOD expression in MHCC97H cells by infection with human MnSOD cDNA-carrying adenoviruses (Additional file 2: Figure S2f). The protein amounts of MnSOD and FoxM1 in MHCC97H cells expressing MnSOD were significantly increased when compared with non-transduced-cells or the vector control group (Fig. 2f, Additional file 2: Figure S2 g). Furthermore, sphere and colony formation capabilities in MHCC97H cells expressing MnSOD were enhanced (Fig. 2g and h, Additional file 2: Figure S2h and i). In addition, the protein amounts of CD133, CD44 and ALDH1 as well as Bmi1, Nanog and Oct4 were elevated (Fig. 2i, Additional file 2: Figure S2j). Luciferase repoter assay showed that the relative luciferase activity of FOXM1 promoter fragment (from − 330 to + 26) that contain E2F1 and Sp1 putative binding sites was enhanced in MHCC97H cells expressing MnSOD compared with non-transduced-cells or the vector control group (Fig. 2j). Taken together, these results suggested MnSOD expression participated in the maintenance of carcinogenicity and stemness by upregulated FoxM1 via an increased binding of E2F1 and Sp1 onto FoxM1 promoter, which was induced by MnSOD constructing a steady flow of H_2_O_2_ originating from mitochondria [16] in HCSLCs from MHCC97H cells.

To determine whether the inhibitory effects of isovitexin on carcinogenicity and stemness involve MnSOD downregulation, HCSLCs were knocked down for MnSOD in the presence or absence of isovitexin, respectively. The results showed the protein amounts of MnSOD and FoxM1 in the MnSOD knockdown plus isovitexin treatment group significantly decreased when compared with MnSOD knockdown or isovitexin treatment single group (Fig. 3a, Additional file 3: Figure S3a). In addition, sphere and colony formation capabilities in the MnSOD knockdown plus isovitexin treatment group were further attenuated (Fig. 3b and c, Additional file 3: Figure S3b and c). Furthermore, the protein amounts of CD133, CD44 and ALDH1 as well as Bmi1, Nanog and Oct4 were reduced by MnSOD knockdown plus isovitexin (Fig. 3d, Additional file 3: Figure S3d). Interestingly, isovitexin cooperated with MnSOD knockdown to inhibit the relative luciferase activity of FOXM1 promoter fragment (from − 330 to + 26) that contain E2F1 and Sp1 putative binding sites (Fig. 3e).

**Fig. 3:** Effects of isovitexin combined with MnSOD shRNA or cDNA on carcinogenicity and stemness in HCSLCs or MHCC97H cells. HCSLCs were transduced with Ad-GFP and Ad-shMnSOD, respectively, incubated with or without isovitexin (ISOV; 10 μM). **a** Immunoblotting performed with anti-MnSOD and anti-FoxM1 antibodies, with β-actin antibodies as a loading control; **b** and **c** Formed spheres and colonies (Scale bar, 200 μm); **d** Immunoblotting for CD133, CD44, ALDH1, Bmi1, Nanog and Oct4; **e** The relative luciferase activity of FOXM1 promoter fragment in HCSLCs transduced with Ad-GFP and Ad-shMnSOD, respectively, in the absence or presence of isovitexin. MHCC97H cells were transduced with Ad-GFP and Ad-MnSOD, respectively, and incubated with or without isovitexin. **f** Immunoblotting performed with anti-MnSOD and anti-FoxM1 antibodies, with β-actin antibodies as a loading control; **g** and **h** Formed spheres and colonies (Scale bar, 200 μm); **i** Immunoblotting for CD133, CD44, ALDH1, Bmi1, Nanog and Oct4; **j** The relative luciferase activity of FOXM1 promoter fragment in MHCC97H cells transduced with Ad-GFP and Ad-MnSOD, respectively, cultured in the absence or presence of isovitexin

We also performed forced expression of MnSOD in MHCC97H cells to explore the mechanism by which isovitexin suppresses carcinogenicity and stemness involves MnSOD downregulation. The results showed that MnSOD overexpression resulted in elevated protein levels of MnSOD and FoxM1 in MHCC97H cells, and nearly abrogated the inhibitory effects of isovitexin (Fig. 3f, Additional file 3: Figure S3e). Furthermore, sphere and colony formation capabilities were enhanced, while the inhibitory effects of isovitexin were declined by MnSOD overexpression (Fig. 3g and h, Additional file 3: Figure S3f and g). Meanwhile, the protein amounts of CD133, CD44 and ALDH1 as well as Bmi1, Nanog and Oct4 were increased, and the inhibitory effects of isovitexin were abolished in MnSOD overexpressing MHCC97H cells (Fig. 3i, Additional file 3: Figure S3h). Furthermore, forced expression of MnSOD in MHCC97H cells could counteract the inhibitory effects of isovitexin on the relative luciferase activity of FOXM1 promoter fragment (from − 330 to + 26) that contain E2F1 and Sp1 putative binding sites (Fig. 3j). Collectively, these results suggested that the inhibitory effects of isovitexin on carcinogenicity and stemness in HCSLCs from MHCC97H cells may be dependent on MnSOD downregulation alleviating H_2_O_2_ flow-mediated E2F1 and/or Sp1 activation [14, 16].

### Isovitexin-associated inhibition of carcinogenicity and stemness is affected by FoxM1 expression alteration in HCSLCs from MHCC97H cells

To assess the role of FoxM1 in sustaining carcinogenicity and stemness, we knocked down FoxM1 in HCSLCs by transduction with FOXM1 shRNA (Additional file 4: Figure S4a). The results showed that FoxM1 knockdown significantly repressed FoxM1 expression in HCSLCs, but had no effect on MnSOD (Fig. 4a, Additional file 4: Figure S4b). In addition, sphere and colony formation capabilities were attenuated in FoxM1 knockdown HCSLCs compared with non-transduced-cells or the vector control (Fig. 4b and c, Additional file 4: Figure S4c and d). Furthermore, the expression levels of CD133, CD44 and ALDH1 as well as Bmi1, Nanog and Oct4 in FoxM1 knockdown HCSLCs were also reduced (Fig. 4d, Additional file 4: Figure S4e).

**Fig. 4:** Effects of FoxM1 shRNA or cDNA transduction on carcinogenicity and stemness in HCSLCs or MHCC97H cells. HCSLCs were transduced with Ad-GFP or Ad-shFoxM1. **a** Immunoblotting performed with anti-MnSOD and anti-FoxM1 antibodies, with β-actin antibodies as a loading control; **b** and **c** Formed spheres and colonies (Scale bar, 200 μm); **d** Immunoblotting for CD133, CD44, ALDH1, Bmi1, Nanog and Oct4 in HCSLCs untreated (Mock), and transduced with Ad-GFP and Ad-shFoxM1, respectively. MHCC97H cells were transduced with Ad-GFP and Ad-FoxM1, respectively. **e** Immunoblotting performed with anti-MnSOD and anti-FoxM1 antibodies, with β-actin antibodies as a loading control; **f** and **g** Formed spheres and colonies (Scale bar, 200 μm); **h** Immunoblotting for CD133, CD44, ALDH1, Bmi1, Nanog and Oct4in MHCC97H cells untreated (Mock), and transduced with Ad-GFP and Ad-FoxM1, respectively

In gain of function experiments, MHCC97H cells were infected with human FOXM1 cDNA-carrying adenoviruses to obtain FoxM1 overexpression (Additional file 4: Figure S4f). Overexpression of FoxM1 notably increased FoxM1 protein levels in MHCC97H cells, but had no effect on MnSOD expression (Fig. 4e, Additional file 4: Figure S4g). In addition, sphere and colony formation capabilities were enhanced in FoxM1 overexpressing MHCC97H cells compared with non-transduced-cells or the vector control (Fig. 4f and g, Additional file 4: Figure S4 h and i). Furthermore, the expression amounts of CD133, CD44 and ALDH1 as well as Bmi1, Nanog and Oct4 (Figure) were elevated in FoxM1 overexpressing MHCC97H cells (Fig. 4h, Additional file 4: Figure S4j). Taken together, these results suggested that elevated FoxM1 was associated with sustaining carcinogenicity and stemness of HCSLCs, which FoxM1 expression alteration did not affect MnSOD expression.

To determine whether the inhibitory effects of isovitexin on carcinogenicity and stemness are dependent on FoxM1 downregulation, HCSLCs expressing FoxM1 shRNA were treated with or without isovitexin. The combination of FoxM1 knockdown with isovitexin was stronger in downregulating the FoxM1 protein compared with FOXM1 knockdown or isovitexin treatment alone, but did not affect the inhibitory effects of isovitexin on MnSOD expression (Fig. 5a, Additional file 5: Figure S5a). In addition, sphere and colony formation capabilities were further reduced in HCSLCs expressing FoxM1 shRNA treated with isovitexin (Fig. 5b and c, Additional file 5: Figure S5b and c). Furthermore, the protein amounts of CD133, CD44 and ALDH1 as well as Bmi1, Nanog and Oct4 were more pronouncedly decreased in HCSLC expressing FoxM1 shRNA treated with isovitexin compared with the FOXM1 knockdown and isovitexin single treatment groups, respectively (Fig. 5d, Additional file 5: Figure S5d).

**Fig. 5:** Effects of isovitexin combined with FoxM1 shRNA or cDNA on carcinogenicity and stemness in HCSLCs or MHCC97H cells. HCSLCs were transduced with Ad-GFP and Ad-shFoxM1, respectively, incubated with or without isovitexin (ISOV; 10 μM). **a** Immunoblotting performed with anti-MnSOD and anti-FoxM1 antibodies, with β-actin antibodies as a loading control; **b** and **c** Formed spheres and colonies (Scale bar, 200 μm); **d** Immunoblotting for CD133, CD44, ALDH1 (D), Bmi1, Nanog and Oct4 amounts in HCSLCs transduced with Ad-GFP and Ad-shFoxM1, respectively, in the absence or presence of isovitexin. MHCC97H cells were transduced with Ad-GFP and Ad-FoxM1, respectively, and incubated with or without isovitexin. **e** Immunoblotting performed with anti-MnSOD and anti-FoxM1 antibodies, with β-actin antibodies as a loading control; **f** and **g** Formed spheres and colonies (Scale bar, 200 μm); **h** Immunoblotting for CD133, CD44, ALDH1, Bmi1, Nanog and Oct4 in MHCC97H cells transduced with Ad-GFP and Ad-FoxM1, respectively, cultured in the absence or presence of isovitexin

To further assess whether the inhibitory effects of isovitexin on carcinogenicity and stemness are dependent on FoxM1 downregulation, FoxM1 overexpressing MHCC97H cells were treated with or without isovitexin. FoxM1 overexpression significantly counterbalanced FoxM1 protein downregulation by isovitexin, but did not affect the inhibitory effects of isovitexin on MnSOD expression compared with FOXM1 knockdown and isovitexin single treatment groups, respectively (Fig. 5e, Additional file 5: Figure S5e). In addition, sphere and colony formation capabilities were enhanced, while the inhibitory effects of isovitexin were lessened by FoxM1 overexpression (Fig. 5f and g, Additional file 5: Figure S5f and g). Furthermore, the protein amounts of CD133, CD44 and ALDH1as well as Bmi1, Nanog and Oct4 were increased, and the inhibitory effects of isovitexin were abolished in FoxM1 overexpressing MHCC97H cells (Fig. 5h, Additional file 5: Figure S5 h). Collectively, these results suggested that the inhibitory effects of isovitexin on carcinogenicity and stemness in HCSLCs may be dependent on FoxM1 downregulation by decreasing MnSOD expression.

### FOXM1 overexpression rescues suppression of MnSOD knockdown plus isovitexin on carcinogenicity and stemness in HCSLCs from MHCC97H cells

To determine whether the inhibitory effects of isovitexin on carcinogenicity and stemness are dependent on MnSOD/FoxM1 axis modulation, HCSLCs expressing MnSOD shRNA and/or treated with or without isovitexin were infected with human FOXM1 cDNA-carrying adenoviruses to achieve FOXM1 overexpression. Analysis of MnSOD and FoxM1 expression levels further demonstrated that overexpression of FoxM1 reversed MnSOD shRNA-mediated FOXM1 downregulation, but did not affect MnSOD protein levels (Fig. 6a, Additional file 6: Figure S6a). Interestingly, overexpression of FoxM1 lessened suppression of MnSOD shRNA on sphere and colony formation capabilities, and reduced the protein amounts of CD133, CD44 and ALDH1 as well as Bmi1, Nanog and Oct4 in HCSLCs (Fig. 6b-d; Additional file 6: Figure S6b-6d). Furthermore, MnSOD and FoxM1 expression levels were analyzed in MnSOD shRNA expressing HCSLCs transduced with FOXM1 cDNA in the presence or absence of isovitexin. Immunoblot showed that overexpression of FoxM1 nearly completely abolished isovitexin- and/or MnSOD-shRNA-mediated FOXM1 downregulation, but did not affect MnSOD protein levels (Fig. 6e, Additional file 6: Figure S6e). In addition, overexpression of FoxM1 significantly decreased isovitexin- and/or MnSOD-shRNA-mediated inhibition of sphere and colony formation capabilities, the protein amounts of CD133, CD44 and ALDH1 as well as Bmi1, Nanog and Oct4 in HCSLCs from MHCC97H cells (Fig. 6f-h, Additional file 6: Figure S6f-h). These findings indicated that blocking the MnSOD/FoxM1 axis is one of the mechanisms required for the inhibition of HCSLC feature by isovitexin.

**Fig. 6:** Isovitexin inhibits HCSLC carcinogenicity and stemness via the MnSOD/FoxM1 axis. HCSLCs or those expressing shMnSOD were transduced with Ad-FoxM1. **a** Immunoblotting performed with anti-MnSOD and anti-FoxM1 antibodies, with β-actin antibodies used as loading control; **b** and **c** Formed spheres and colonies (Scale bar, 200 μm); **d** Immunoblotting for CD133, CD44, ALDH1, Bmi1, Nanog and Oct4 in HCSLCs untreated (Mock), and transduced with Ad-shMnSOD and/or Ad-FoxM1. HCSLCs expressing shMnSOD were transduced with Ad-FoxM1 and incubated with or without isovitexin (ISOV; 10 μM). **e** Immunoblotting performed with anti-MnSOD and anti-FoxM1 antibodies, with β-actin antibodies as a loading control; **f** and **g** Formed spheres and colonies (Scale bar, 200 μm); **h** Immunoblotting for CD133, CD44, ALDH1, Bmi1, Nanog and Oct4 in MHCC97H cells transduced with Ad-shMnSOD and/or Ad-FoxM1 and incubated in the absence or presence of ISOV

### Co-administration of isovitexin and thiostrepton cooperated with MnSOD knockdown to repress xenograft growth of HCSLCs in nude mice

To determine the role of MnSOD/FoxM1 axis modulation in isovitexin-associated inhibition or xenograft tumor growth in vivo, mice bearing HCSLC tumors were orally treated every 2 days with 200 μl of vehicle, 10 mg/kg isovitexin or 5 mg/kg thiostrepton (specific inhibitor of FOXM1), or intratumorally injected with adenovirus expressing MnSOD shRNA (once a week) or combination of isovitexin plus thiostrepton and adenovirus, respectively. We found that isovitexin, thiostrepton as a positive control for FoxM1 inhibition and MnSOD knockdown alone resulted in tumor growth inhibition (Fig. 7a-c). Addition of thiostrepton plus MnSOD knockdown and isovitexin resulted in significantly stronger anti-tumor activity in HCSLC xenograft nude mouse models compared with either agent alone (Fig. 7a-c). MnSOD and FoxM1 expression levels assessed by immunohistochemistry in tumor tissues further demonstrated that isovitexin alone had minimal effects on MnSOD and FoxM1 protein expression levels, modest decreases of MnSOD and FoxM1 expression levels in MnSOD knockdown tumors (Fig. 7d). Thiostrepton alone had minimal effects on FoxM1 expression, but did not alter MnSOD protein amounts (Fig. 7d). Meanwhile, isovitexin/thiostrepton combined with MnSOD knockdown significantly reduced the protein expression levels of MnSOD, CD133 and FoxM1 in HCSLC xenograft tumors (Fig. 7d). These findings indicated that MnSOD and FoxM1 protein downregulation might be involved in isovitexin associated reduction of xenograft tumor growth of HCSLCs in nude mice.

**Fig. 7:** Co-administration of isovitexin/thiostrepton and MnSOD knockdown cooperatively suppress xenograft tumor growth of HCSLCs from MHCC97H cells in nude mice. **a** Xenograft tumors were photographed after treatment with vehicle, 10 mg/kg isovitexin or 5 mg/kg thiostrepton, intratumoral injection of adenovirus expressing MnSOD shRNA (once a week), or combination of isovitexin/thiostrepton plus adenovirus for 21 days in nude mice. **b** Tumor volumes in the vehicle control, isovitexin, thiostrepton, MnSOD shRNA, and combination treatment groups. Data are mean ± SD (*n* = 6); *P* < 0.05 indicated statistical significance. ^*^Vehicle control. ^#^Combination treatment group. **c** Xenograft tumor weights in the vehicle control, isovitexin, thiostrepton, MnSOD shRNA, and combination treatment groups. Data are mean ± SD (*n* = 6); *P* < 0.05 indicated statistical significance. ^*^Vehicle control. ^#^Combination treatment group. **d** Upper panel, H&E staining of xenograft tumors in the vehicle control, isovitexin, thiostrepton, MnSOD shRNA and combination treatment groups; middle panel, representative immunohistochemical data for MnSOD in the vehicle control, isovitexin, thiostrepton, MnSOD shRNA and combination treatment groups (magnification, × 400); lower panel, representative immunohistochemical data for FoxM1 in the vehicle control, isovitexin, thiostrepton, MnSOD shRNA and combination treatment groups (magnification, × 400)

### The MnSOD/FoxM1 axis is a novel target for isovitexin-associated inhibition of carcinogenicity and stemness in HCSLCs

To assess the catholicity of FoxM1 upregulation by MnSOD overexpression in sustaining carcinogenicity and stemness in HCSLCs, we selected two additional established hepatic carcinoma cell lines, including HepG2 and SMMC-7721 cells, to compare MnSOD and FoxM1 expression levels, sphere and colony formation capabilities and protein expression levels of CD133, CD44 and ALDH1 between HepG2 or SMMC-7721 cells and the corresponding HCSLCs. Substantially increased MnSOD and FoxM1 amounts, sphere and colony formation capabilities and protein expression levels of CD133, CD44 and ALDH1 were observed in HCSLCs compared with the parent HepG2 or SMMC-7721 cells (Fig. 8a-d). These results suggested that FoxM1 upregulation by MnSOD overexpression was not specific to the cell type originating HCSLCs. More importantly, isovitexin also reduced the amounts of MnSOD and FoxM1 expression in HCSLCs from HepG2 and SMMC-7721 cells (Fig. 8e). Conclusively, these results suggested that the MnSOD/FoxM1 axis might be a novel target for isovitexin-associated inhibition on carcinogenicity and stemness in HCSLCs.

**Fig. 8:** The MnSOD/FoxM1 axis is a novel target for isovitexin-associated inhibition of carcinogenicity and stemness in HCSLCs from HepG2 and SMMC-7721 cells **a** Immunoblotting for MnSOD and FoxM1 expression levels in HepG2 and SMMC-7721 cells and respective HCSLCs, with β-actin antibodies as a loading control; **b** and **c** Sphere and colony formation rates in HepG2 and SMMC-7721 cells and respective HCSLCs. **d** Immunoblotting for determining CK133, CD44 and ALDH1 expression level in HepG2 and SMMC-7721 cells and respective HCSLCs, with β-actin as an internal control. Data are mean ± SD (*n* = 3); *P* < 0.05 indicated statistical significance. ^*^ HepG2 cells. ^#^SMMC-7721 cells. **e** Immunoblotting for assessing MnSOD and FoxM1 expression levels in HCSLCs from HepG2 and SMMC-7721 cells incubated with or without isovitexin (ISOV; 10 μM). Data are mean ± SD (*n* = 3); *P* < 0.05 indicated statistical significance. ^*^ Vehicle control in HCSLCs from HepG2 cells. ^#^Vehicle control in HCSLCs from SMMC-7721 cells. **f** Schematic diagram of the mechanism underlying isovitexin inhibits HCSLC carcinogenicity and stemness via the MnSOD/FoxM1 axis. Isovitexin effectually inhibited carcinogenicity and stemness in HCSLCs by downregulating FoxM1 likely through preventing MnSOD overexpression induced mitochondrial H_2_O_2_-mediated an increased binding of E2F1 and Sp1 onto FoxM1 promoter

## Discussion

The present study demonstrated that carcinogenicity and stemness in HCSLCs are inhibited by isovitexin through MnSOD/FoxM1 axis modulation. These results highlight the notion that modulating elevated MnSOD that upregulates FoxM1 through an increased binding of E2F1 and Sp1 onto FoxM1 promoter is a novel way for suppressing carcinogenicity and stemness in HCSLCs to treat human hepatic carcinoma. Increasing evidence indicates that hepatic carcinoma possesses CSLCs, which would significantly influence the design and evaluation of novel targeted therapeutic agents for human hepatic carcinoma.

Hart et al. [16] reported that MnSOD generates stronger oxidant H_2_O_2_ than superoxide anion radicals, thereby regulating mitochondria-driven signaling in the cell, and MnSOD suppression caused by H_2_O_2_-associated signaling leads to metabolic collapse and cell death in breast cancer MDA-MB-231 cells. Recent studies from our and other Laboratories have shown that MnSOD overexpression is associated with CSLC functions and characteristics [15, 30–33]. In the present study, parallels between elevated MnSOD amounts and enhanced sphere and colony formation capabilities, a high expression of stemness-related markers as well as an increased percentage of CD133^+^ cells with LCSLC characteristics were observed by comparison of HCSLCs with respective parental cells. In MHCC97H cells, MnSOD overexpression potentiated sphere and colony formation capabilities and increased the protein expression levels of stemness-related markers. Conversely, MnSOD knockdown in HCSLCs reduced sphere and colony formation capabilities as well as the protein amounts of stemness-related markers. Therefore, MnSOD may be involved in the promotion and maintenance of carcinogenicity and stemness in HCSLCs.

A study by Chen et al. showed that FoxM1expression level alteration does not change MnSOD expression, whereas MnSOD overexpression significantly increases FoxM1 expression levels by releasing the E2F1 and Sp1 transcription factors [14]. Our recent study also obtained similar results in lung CSLCs [15]. Consistent with those findings, we here showed that alteration of MnSOD expression markedly affected FoxM1 expression and the relative luciferase activity of FOXM1 promoter fragment (from − 330 to + 26) that contain E2F1 and Sp1 putative binding sites, whereas FOXM1 expression alteration did not affect MnSOD expression in HCSLCs from MHCC97H. Nonetheless, we also provided experimental evidence that FOXM1 overexpression could rescue suppression of MnSOD knockdown on HCSLC functions and characteristics. Accordingly, the MnSOD/FoxM1 axis might facilitate and maintain HCSLC characteristics and stemness.

Isovitexin causes apoptosis and autophagy in various cancer cells through regulation of apoptosis- and autophagy-associated proteins, and signaling molecules have been investigated in many experimental systems in vitro and in vivo [23–29]. Fructus Viticis total flavonoids containing isovitexin effectively inhibit CSLC characteristics in H446 cells [26]. However, few antineoplastic effects targeting HCSLCs inhibition by isovitexin treatment have been examined. In the current study, we demonstrated that isovitexin substantially decreased sphere and colony formation abilities, protein amounts of stemness-related markers as well as CD133^+^ cell subpopulation in HCSLCs in vitro. Orally administered isovitexin also showed powerful inhibitory effects on xenograft tumor growth of HCSLCs in vivo, which reflects the potential clinical value of isovitexin and the urgent necessity to further perform clinical trials for confirmation. More importantly, isovitexin showed significant therapeutic effects on human hepatic carcinoma by targeting HCSLCs via modulation of the MnSOD/FoxM1 signaling axis. The role of the MnSOD/FoxM1 signaling axis as a direct elimination target for carcinogenicity and stemness in hepatic carcinomas has been less appreciated. In the present study, we demonstrated that isovitexin effectually reduced the relative luciferase activity of FOXM1 promoter fragment (from − 330 to + 26) that contain E2F1 and Sp1 putative binding sites, which was enhanced by MnSOD knockdown and attenuated by MnSOD overexpression. Together, our results suggest that isovitexin effectually inhibited carcinogenicity and stemness in HCSLCs by downregulating FoxM1 likely through preventing MnSOD overexpression induced mitochondrial H_2_O_2_-mediated an increased binding of E2F1 and Sp1 onto FoxM1 promoter (Fig. 8f). Consistent with these results, MnSOD and associated FoxM1 upregulation have recently been shown to participate in controlling carcinogenicity and malignancy by converting H460 cells to suspension sphere growth of the CSLC phenotype [15] and promoting cell migration and invasion [14]. However, how isovitexin inhibits FoxM1 induced by abnormal expression of MnSOD and in what way MnSOD modulates FoxM1 expression require further investigation.

## Conclusions

In summary, the current study provides a novel insight into suppression of isovitexin on HCSLC properties and tumor growth through blocking of the MnSOD/FoxM1 axis. These findings suggest isovitexin as a promising therapeutic agent for hepatic carcinoma patients. In the future, the safety and efficacy of isovitexin as a novel agent for hepatic carcinoma patients will be evaluated in clinical studies.

## Additional files

Additional file 1: **Figure S1.** Isovitexin inhibits carcinogenicity and stemness in HCSLCs. Quantitation of (a) MnSOD and FoxM1 protein expressions; (b) Spheroid formation; (c) Colony formation; (d) CD133, CD44, ALDH1, Bmi1, Nanog and Oct4 proteins; (e) CD133^+^ cell population in MHCC97H cells and HCSLCs. Data are mean ± SD (*n* = 3); *P* < 0.05 indicated statistical significance. ^*^MHCC97H cells. (f) HCSLCs (1 × 10^3^ cells) or MHCC97H cells (1 × 10^5^ cells) were subcutaneously injected into male BALB/c-nu mice. After 2 months, xenograft tumors were photographed (f1). The column graphs represent tumor volumes (f2) and weights (f3). H&E staining showed similar histological features, but CD133 protein levels elevated, as examined by immunohistochemisty for xenograft tumors from HCSLCs and MHCC97H cells (f4). Data are mean ± SD (*n* = 6); *P* < 0.05 indicated statistical significance. ^*^Xenograft tumors of MHCC97H cells. (g) Decreased the amounts of MnSOD and FoxM1 in HCSLCs from MHCC97H cells following treatment with isovitexin (ISOV: 5.0, 10.0 and 20.0 μM). Isovitexin induced reduction of spheroid formation (h), colony formation (i), and protein amounts of CD133, CD44, ALDH1 and Bmi1, Nanog and Oct4 (j) CD133^+^ cell population (k) in HCSLCs. Data are mean ± SD (*n* = 3); *P* < 0.05 indicated statistical significance. ^*^vehicle control; ^#^5.0 μM isovitexin (ISOV). (l1) Xenograft tumors were photographed after treatment with vehicle or isovitexin (10, 20 and 40 mg/kg body weight) for 21 days in nude mice. (l2) Xenograft weights in the vehicle control and isovitexin treated groups. Data are mean ± SD (*n* = 6); *P* < 0.05 indicated statistical significance. ^*^Vehicle control. ^#^Isovitexin (10 mg/kg). (l3) H&E staining and immunohistochemisty with CD133 antibody of xenograft tumors in the vehicle control and isovitexin treatment groups. (TIF 9542 kb)

Additional file 2: **Figure S2.** Effects of MnSOD shRNA or cDNA transduction on carcinogenicity and stemness in HCSLCs or MHCC97H cells. (a) MnSOD knockdown decreased sphere formation in HCSLCs from MHCC97 cells. Data are mean ± SD (*n* = 3); *P* < 0.05 indicated statistical significance. ^*^Transduced with Ad-GFP. Representative immunofluorescent images are shown (magnification: × 200). Quantitation of (b) MnSOD and FoxM1 protein expressions; (c and d) Formed spheres and colonies; (e) CD133, CD44 and ALDH1, Bmi1, Nanog and Oct4 protein expressions; (f) MnSOD overexpression in MHCC97 cells. Representative immunofluorescent images are shown (magnification: × 200). Quantitation of (g) MnSOD and FoxM1 protein expressions; (h and i) Formed spheres and colonies; (j) CD133, CD44, ALDH1, Bmi1, Nanog and Oct4 protein expressions in MHCC97H cells untreated (Mock), and transduced with Ad-GFP and Ad-MnSOD, respectively. Data are mean ± SD (*n* = 3); *P* < 0.05 indicated statistical significance. ^*^untreated or transduced with Ad-GFP control. (TIF 4591 kb)

Additional file 3: **Figure S3.** Effects of isovitexin combined with MnSOD shRNA or cDNA on carcinogenicity and stemness in HCSLCs or MHCC97H cells. HCSLCs were transduced with Ad-GFP and Ad-shMnSOD, respectively, incubated with or without isovitexin (ISOV; 10 μM). Quantitation of (a) MnSOD and FoxM1 protein expressions; (b and c) Formed spheres and colonies; (d) CD133, CD44, ALDH1, Bmi1, Nanog and Oct4 protein expressions in HCSLCs transduced with Ad-GFP and Ad-shMnSOD, respectively, in the absence or presence of isovitexin. MHCC97H cells were transduced with Ad-GFP and Ad-MnSOD, respectively, and incubated with or without isovitexin. Quantitation of (e) MnSOD and FoxM1 protein expressions; (f and g) Formed spheres and colonies; (h) CD133, CD44, ALDH1, Bmi1, Nanog and Oct4 protein expressions in MHCC97H cells transduced with Ad-GFP and Ad-MnSOD, respectively, cultured in the absence or presence of isovitexin. Data are mean ± SD (*n* = 3); *P* < 0.05 indicated statistical significance. ^*^Ad-GFP transduced control; ^#^ Ad-GFP transduction and treated with 10 μM isovitexin (ISOV). (TIF 2436 kb)

Additional file 4: **Figure S4.** Effects of FoxM1 shRNA or cDNA transduction on carcinogenicity and stemness in HCSLCs or MHCC97H cells. (a) FoxM1 knockdown decreased sphere formation in HCSLCs and MHCC97H cells. Data are mean ± SD (*n* = 3); *P* < 0.05 indicated statistical significance. ^*^Transduced with Ad-GFP. Representative immunofluorescent images are shown (magnification: × 200). Quantitation of (b) MnSOD and FoxM1 protein expressions; (c and d) Formed spheres and colonies; (e) CD133, CD44, ALDH1, Bmi1, Nanog and Oct4 protein expressions in HCSLCs untreated (Mock), and transduced with Ad-GFP and Ad-shFoxM1, respectively. (f) FoxM1 overexpression increased sphere formation in MHCC97H cells. Data are mean ± SD (*n* = 3); *P* < 0.05 indicated statistical significance. ^*^Transduced with Ad-GFP. Representative immunofluorescent images are shown (magnification: × 200). Quantitation of (g) MnSOD and FoxM1 protein expressions; (h and i) Formed spheres and colonies; (j) CD133, CD44, ALDH1, Bmi1, Nanog and Oct4 protein expressions in MHCC97H cells untreated (Mock), and transduced with Ad-GFP and Ad-FoxM1, respectively. Data are mean ± SD (*n* = 3); *P* < 0.05 indicated statistical significance. ^*^untreated or transduced with Ad-GFP control. (TIF 3856 kb)

Additional file 5: **Figure S5.** Effects of isovitexin combined with FoxM1 shRNA or cDNA on carcinogenicity and stemness in HCSLCs or MHCC97H cells. HCSLCs were transduced with Ad-GFP and Ad-shFoxM1, respectively, incubated with or without isovitexin (ISOV; 10 μM). Quantitation of (a) MnSOD and FoxM1 protein expressions; (b and c) Formed spheres and colonies; (d) CD133, CD44, ALDH1, Bmi1, Nanog and Oct4 protein expressions in HCSLCs transduced with Ad-GFP and Ad-shFoxM1, respectively, in the absence or presence of isovitexin. MHCC97H cells were transduced with Ad-GFP and Ad-FoxM1, respectively, and incubated with or without isovitexin. Quantitation of (e) MnSOD and FoxM1 protein expressions; (f and g) Formed spheres and colonies; (h) CD133, CD44, ALDH1, Bmi1, Nanog and Oct4 protein expressions in MHCC97H cells transduced with Ad-GFP and Ad-FoxM1, respectively, cultured in the absence or presence of isovitexin. Data are mean ± SD (*n* = 3); *P* < 0.05 indicated statistical significance. ^*^Ad-GFP transduced control; ^#^ Ad-GFP transduction and treated with 10 μM isovitexin (ISOV). (TIF 2422 kb)

Additional file 6: **Figure S6.** Isovitexin inhibits HCSLC carcinogenicity and stemness via the MnSOD/FoxM1 axis. HCSLCs or those expressing shMnSOD were transduced with Ad-FoxM1. Quantitation of (a) MnSOD and FoxM1 protein expressions; (b and c) Formed spheres and colonies; (d) CD133, CD44, ALDH1 (D), Bmi1, Nanog and Oct4 protein expressions in HCSLCs untreated (Mock), and transduced with Ad-shMnSOD and/or Ad-FoxM1. Data are mean ± SD (*n* = 3); *P* < 0.05 indicated statistical significance. ^*^ Untreated control; ^#^ Transduced with Ad-shMnSOD. HCSLCs expressing shMnSOD were transduced with Ad-FoxM1 and incubated with or without isovitexin (ISOV; 10 μM). Quantitation of (e) MnSOD and FoxM1 protein expressions; (f and g) Formed spheres and colonies; (h) CD133, CD44, ALDH1 (D), Bmi1, Nanog and Oct4 protein expressions in MHCC97H cells transduced with Ad-shMnSOD and/or Ad-FoxM1 and incubated in the absence or presence of ISOV. Data are mean ± SD (*n* = 3); *P* < 0.05 indicated statistical significance.^*^Transduced with Ad-shMnSOD; ^#^ Transduced with Ad-shMnSOD and treated with 10 μM isovitexin (ISOV). (TIF 2481 kb)

## Data Availability

The datasets used and/or analysed during the current study are available from the corresponding author on reasonable request.

## Abbreviations

ANOVA: Analysis of variance
CSC-CM: Cancer stem cell conditioned medium
FoxM1: Forkhead box M1
FVTF: Fructus Viticis total flavonoids
H_2_O_2_: Hydrogen peroxide
HCSLCs: Hepatic carcinoma stem-like cells
LSD: Least significant difference
MnSOD: Manganese superoxide dismutase
SD: Standard deviation
SDS-PAGE: Sodium dodecyl sulfate polyacrylamide gel electrophoresis
